# Progressive Rapid Atherosclerotic Plaque Formation and Early Stent re‐Stenosis in an Untreated CLL Patient; A Case Report

**DOI:** 10.1002/ccr3.72619

**Published:** 2026-04-26

**Authors:** Mohammad Shojae, Hosseinali Rostamipour, Aref Ghanaatpisheh, Sepehr Ramezanipour, Nikta Heidari

**Affiliations:** ^1^ Cardiology Department Jahrom University of Medical Sciences Jahrom Iran; ^2^ Department of Internal Medicine Jahrom University of Medical Sciences Jahrom Iran; ^3^ Student Research Committee Jahrom University of Medical Sciences Jahrom Iran; ^4^ Student Research Committee Fasa University of Medical Sciences Fasa Iran

**Keywords:** angiography, atherosclerosis, CLL, NSTEMI

## Abstract

A 66 year‐old male with a history of hypertension and poor follow‐up for chronic lymphocytic leukemia (CLL) experienced two episodes of non‐ST elevation myocardial infarction (NSTEMI) within a 6 month period. Initial coronary angiography showed two‐vessel disease, and percutaneous coronary intervention (PCI) was performed on the left anterior descending artery (LAD). Six months later, repeat angiography revealed rapid progression to three‐vessel disease, including in‐stent restenosis and new severe lesions, which required urgent coronary artery bypass grafting (CABG). Laboratory tests indicated persistent leukocytosis, with white blood cell (WBC) counts increasing from 38.6 × 10^3^/μL to 75.7 × 10^3^/μL. This case highlights a rare but clinically significant association between CLL and accelerated coronary artery disease (CAD), suggesting potential mechanisms such as leukocyte aggregation, endothelial injury, and amyloid deposition contributing to rapid atherosclerosis. The findings underscore the importance of thorough cardiac evaluation in CLL patients and the need for further research into the underlying mechanisms and optimal treatment strategies for this high‐risk group.

## Key Clinical Message

This case of rapid, severe coronary artery progression in a patient with CLL highlights a critical hematologic‐cardiac link. It underscores the necessity for vigilant cardiac surveillance in CLL patients, especially those with elevated and rising white blood cell counts, to mitigate the risk of accelerated atherosclerosis and major adverse cardiac events.

## 1 Introduction

The rapid progression of atherosclerotic plaque in coronary arteries is a critical concern in cardiovascular health, characterized by significant changes in plaque morphology and stability within short time frames. This phenomenon is often defined by a greater than 10% reduction in the diameter of existing stenosis or the development of new lesions leading to total occlusion within months. Recent studies have identified several predictors of this rapid progression, including elevated levels of inflammatory markers such as C‐reactive protein (CRP) and endothelin, which are associated with increased plaque instability and vulnerability [1, 2]. Additionally, traditional cardiovascular risk factors do not consistently correlate with rapid disease progression, suggesting that other mechanisms, such as genetic predispositions and inflammatory responses, or also cancers such as CLL play a significant role in accelerating atherosclerosis [3].

Over the past two decades, case reports have described uncommon instances of CLL infiltration into coronary arteries, highlighting its potential contribution to coronary artery disease [4, 5].

CLL is a common type of leukemia, primarily affecting the elderly population. It is characterized by the accumulation of mature‐appearing neoplastic lymphocytes in lymphoid tissues, bone marrow, and peripheral blood vessels. The clinical presentation of CLL varies widely, ranging from asymptomatic cases, often diagnosed incidentally through elevated lymphocyte counts in peripheral blood, to those with constitutional symptoms. The diagnosis of CLL is confirmed through blood smears, complete blood counts, and the detection of circulating B‐lymphocytes with clonal populations expressing the CD5 antigen [6].

CLL is among the most prevalent hematological malignancies (HM) in older individuals. Despite its high prevalence in this population, population‐based studies have identified cardiovascular diseases, such as myocardial infarction (MI), as the second leading cause of death in these patients [7]. Additionally, rare reports in the medical literature have described coronary artery occlusion and cardiac infiltration associated with CLL [7, 8].

Here, we report a 66‐year‐old man with untreated CLL who developed two non–ST‐segment elevation myocardial infarctions (NSTEMIs) within 6 months, accompanied by rapid multivessel atherosclerotic progression and early in‐stent restenosis of the left anterior descending artery (LAD). This case underscores the potential interplay between CLL‐related hematologic abnormalities and accelerated coronary disease and highlights the need for heightened cardiovascular vigilance in patients with hematologic malignancies.

## 2 Case History and Examination

A 66‐year‐old man with a 10‐year history of hypertension and a 2 year history of CLL presented to the Emergency Department of Peymanieh Hospital, Jahrom, Iran, with sudden‐onset, compressive chest pain and dyspnea lasting approximately 14 h. At the time of his CLL diagnosis, he had been evaluated by a hematologist and did not meet criteria for treatment, so a watch‐and‐wait strategy was adopted. The patient subsequently did not adhere to regular hematologic follow‐up by personal choice.

The current episode of chest pain was similar in character and intensity to symptoms he had experienced during a prior NSTEMI 6 months earlier.

### 2.1 First NSTEMI (Six Months Prior to Index Admission)

Six months before the present admission, the patient had presented to our center with prolonged chest pain of more than 8 h. An initial 12‐lead electrocardiogram (ECG) (Figure 1) showed changes consistent with non–ST‐segment elevation acute coronary syndrome. Serial cardiac troponin measurements were elevated, confirming the diagnosis of NSTEMI. The patient was treated with standard guideline‐directed medical therapy, including antiplatelet agents and anti‐ischemic medications (exact regimen available in Table 1, if you wish to include it).

**FIGURE 1:** (ECG of first chest pain at ED).

**TABLE 1:** Summary of Lab data during admission.

First admission		Second admission	
Lab data factor	Lab data factor	Lab data factor	Lab data factor
WBC	38.6 × 10^3^/Mic	WBC	75.7 × 10^3^/Mic
RBC	5.45 × 10^6^/Mic	RBC	5.05 × 10^6^/Mic
HB	14.7 g/dL	HB	13.1 g/dl
HCT	43.80%	HCT	39.40%
MCV	80.37 f	MCV	78.02 f
MCH	26.97 Pg	MCH	25.94 Pg
MCHC	33.56 g/dL	MCHC	33.25 g/dL
PLT	151 × 10^3^/Mic	PLT	171 × 10^3^/Mic
BUN	13 mg/dL	BUN	12 mg/dL
Creat	0.7 mg/dL	Creat	1.1 mg/dL
Na	136 mEq/L	Na	136 mEq/L
K	4 mEq/L	K	3.9 mEq/L
Troponin	Positive	Troponin	Positive
PT	12.8 Sec	PT	12.6 Sec
PTT	26 Sec	PTT	26 Sec
INR	1.03	INR	1
HDL	26	—	—
LDL	47.6	—	—
Cholesterol	102	—	—
TG	147	—	—

Transthoracic echocardiography demonstrated a left ventricular ejection fraction (LVEF) of 45% with mild tricuspid regurgitation. Laboratory evaluation revealed leukocytosis with a white blood cell (WBC) count of 38.6 × 10^3^/μL and a platelet count of 151 × 10^3^/μL, while other routine parameters are summarized in Table 1. The WBC count was markedly above the normal range.

Coronary angiography (Video S1) via right radial access, performed by an experienced interventional cardiologist, revealed significant atherosclerotic plaques in the mid and distal segments of the LAD and moderate lesions in the right coronary artery (RCA), consistent with two‐vessel coronary artery disease. The LAD lesion was deemed the culprit, and percutaneous coronary intervention (PCI) with stent implantation (details of stent type and size should be specified if available) was performed on the LAD with a good angiographic result.

Following stabilization, the patient was referred for hematology consultation due to persistent leukocytosis, which led to the confirmation of CLL by blood counts, peripheral smear, and immunophenotyping. He was discharged with a combined cardiac and hematologic follow‐up plan and was advised to adhere to regular outpatient visits.

### 2.2 Second Episode of NSTEMI

Six months after the initial NSTEMI, the patient re‐presented with recurrent chest pain and dyspnea. ECG (Figure 2) again showed findings compatible with NSTEMI, and troponin levels were positive. Laboratory tests revealed a further rise in WBC count to 75.7 × 10^3^/μL and a hemoglobin level of 13.1 g/dL; additional laboratory data are summarized in (Table 1).

**FIGURE 2:** (ECG of second Episode of NSTEMI).

Repeat echocardiography, performed by a different cardiologist, showed a preserved LVEF of 55% with no new significant valvular abnormalities. Emergent coronary angiography (Video S2), performed by the same interventional cardiologist who managed the first event, demonstrated marked progression of coronary artery disease. There were now severe stenoses in the posterior descending artery (PDA), RCA, left circumflex artery (LCX), obtuse marginal branches, and diagonal branches, along with significant in‐stent restenosis of the previously treated LAD segment. Overall, the angiographic findings were consistent with new‐onset three‐vessel disease.

In view of the extent and severity of the disease, and the presence of early in‐stent restenosis in the LAD, the heart team recommended urgent coronary artery bypass grafting (CABG). Due to the complexity of his coronary anatomy and the need for advanced cardiac surgical care, the patient was transferred to a tertiary referral center in Shiraz, Iran, for further management and surgical intervention.

## 3 Discussion

This case illustrates a rare but clinically important scenario of rapid multivessel atherosclerotic progression and early in‐stent restenosis in a patient with untreated CLL. The progression from two‐vessel disease with single‐vessel PCI to extensive three‐vessel disease, including restenosis of the LAD stent, occurred within only 6 months and was paralleled by a substantial rise in leukocyte count. This temporal association raises the possibility that CLL‐related pathophysiological mechanisms may have contributed to accelerated coronary disease beyond traditional cardiovascular risk factors.

Cardiac involvement, including cardiac infiltration and coronary syndromes, is an exceptionally rare occurrence in CLL and has been documented in only a limited number of case reports or reviews. The present case provides an opportunity to summarize and critically evaluate the spectrum of cardiac, coronary involvement, and progressive atherosclerosis in CLL populations.

In 1981, Schwartz and colleagues investigated the involvement of various organs in patients with leukemia. Their findings revealed cardiac involvement in 64% of the studied population, with most cases being asymptomatic. However, follow‐up studies conducted 30 years later indicated that among symptomatic cases, the most prevalent manifestations included heart failure, cardiac arrest, and arrhythmias [9, 10].

Similarly to our case, Assiri et al. (2004) reported an 83 year‐old male with a 10 year history of CLL who presented with hypotension and dyspnea. Unfortunately, the patient died shortly after admission. However, autopsy findings revealed significant observations, including evidence of myocardial infarction in the inferolateral wall of the left ventricle and severe coronary artery atherosclerosis. Additionally, leukemic infiltration was identified in the walls of the coronary arteries [4]. Another case involving CLL with coronary artery involvement was described by Bennet et al., who reported on a 72 year‐old male with CLL. This patient was admitted with symptoms of cough and diarrhea and was initially treated for sepsis and pneumonitis. On the 12th day of hospitalization, the patient developed chest pain. Subsequent investigations, including positive troponin levels and ECG changes, indicated acute coronary syndrome affecting the anterolateral region of the left ventricle [7]. Further diagnostic imaging with cardiac magnetic resonance imaging (MRI) and thoracic computed tomography (CT) revealed a mediastinal mass exerting pressure on the left circumflex (LCX) artery, leading to myocardial ischemia in the affected region.

To explain how myocardial infarction might be related to CLL, several possible mechanisms have been proposed, as discussed in a similar case report by Htet et al., which examined renal and cardiac complications in CLL [11]. These possible mechanisms primarily focus on the role of elevated WBC counts, as their case reported acute coronary syndrome and positive troponin levels following a significant increase in peripheral WBC counts, a pattern also observed in our case.

Several mechanisms may explain how CLL contributes to rapid coronary disease progression. Elevated WBC counts may predispose patients to coronary thrombosis or accelerate atherosclerotic plaque formation, a pattern consistent with the rapid plaque progression seen in our patient. Leukocyte aggregation may further activate coagulation pathways or induce endothelial injury, promoting a pro‐thrombotic state, while amyloid deposition—reported in some CLL patients—may infiltrate vascular structures and contribute to ischemic events [12, 13].

Chronic inflammation and endothelial activation also represent important pathways. CLL is characterized by immune dysregulation and cytokine release, and elevated inflammatory markers such as CRP and IL‐6 are associated with adverse cardiovascular outcomes and rapid coronary progression, including in NSTE‐ACS [5, 14]. This inflammatory milieu may amplify endothelial dysfunction, promote plaque instability, and accelerate neointimal hyperplasia after stent placement. Severe leukocytosis, as observed in this case, can increase blood viscosity, enhance leukocyte–endothelium interactions, and contribute to microvascular obstruction and thrombosis. Prior reports of “leukemic ischemia” support the role of excessive leukocyte burden in worsening coronary lesions [15]. The doubling of WBC count between the two NSTEMI episodes aligns with this mechanism. Amyloid involvement remains another consideration, as CLL may coexist with AL or secondary amyloidosis, which can cause intramural coronary narrowing and impaired vasoreactivity [16]. Although not confirmed histologically in our patient, amyloid‐related vascular dysfunction cannot be excluded. Finally, conventional contributors to restenosis such as suboptimal stent expansion, neoatherosclerosis, clopidogrel resistance, dyslipidemia, or medication nonadherence may act alongside CLL‐related biologic factors [1]. Limited data on stent characteristics, lipid levels, and adherence prevent complete distinction between these overlapping influences in this case.

## 4 Limitations

Our report has several limitations. First, no intravascular imaging (IVUS/OCT) was performed to characterize stent expansion, neointimal proliferation, or neoatherosclerosis, which limits mechanistic insight into early in‐stent restenosis. Second, comprehensive data on lipid profile, antiplatelet adherence, and genetic or functional testing for antiplatelet resistance were not available. Third, there was no histopathologic confirmation of leukemic or amyloid infiltration in the coronary arteries or myocardium. Finally, as a single case report, causal relationships between CLL and accelerated coronary disease cannot be definitively established.

## 5 Conclusion

This case highlights the importance of integrating comprehensive cardiovascular assessment into the routine care of patients with CLL, as emerging evidence including the rapid progression from two to three‐vessel coronary artery disease with early in‐stent restenosis observed here suggests a potential link between CLL‐related inflammatory and hematologic abnormalities and accelerated atherosclerosis. Although direct leukemic infiltration of the coronary arteries was not demonstrated, the temporal association between rising leukocytosis and angiographic deterioration underscores the need for heightened vigilance, particularly in patients with pre‐existing coronary disease.

Given the rarity yet clinical significance of cardiac complications in CLL, further research is needed to clarify the mechanisms involved whether leukocyte aggregation, elevated counts, amyloid deposition, or other pathways and to identify high‐risk subgroups. Prospective studies will be essential to refine diagnostic protocols and develop targeted preventive and therapeutic strategies that address the unique cardiovascular risks faced by patients with CLL.

## Author Contributions

**Mohammad Shojae:** conceptualization, investigation, project administration, resources, supervision, validation, writing – review and editing. **Hosseinali Rostamipour:** conceptualization, data curation, investigation, resources, supervision, validation. **Aref Ghanaatpisheh:** conceptualization, investigation, project administration, supervision, writing – original draft, writing – review and editing. **Sepehr Ramezanipour:** writing – original draft, writing – review and editing. **Nikta Heidari:** methodology, writing – original draft.

## Funding

The authors have nothing to report.

## Consent

Written informed consent was obtained from the patient for the publication of this case report and all accompanying images. The patient specifically requested that their name and any directly identifying personal details not be included in this publication. The consent form is held by the authors and is available for review by the Editor‐in‐Chief of this journal. The patient's family was also informed of this publication and provided their approval.

## Conflicts of Interest

The authors declare no conflicts of interest.

## Supporting information


**Video S1:** First admission coronary angiography demonstrated significant atherosclerotic plaques in the LAD and RCA.

**Video S2:** Second admission, coronary angiography demonstrated PDA, RCA, LCX stenosis, and in‐stent restenosis of the previously treated LAD segment.

## Data Availability

All clinical data and imaging materials supporting the findings of this case report are original. The data have not been published previously and are presented here for the first time. Due to patient privacy and ethical considerations, the underlying raw clinical data are not publicly available but can be provided in de‑identified form by the corresponding author upon reasonable request and with institutional approval.
